RETRACTED

# Application of the PBL Model Based on Deep Learning in Physical Education Classroom Integrating Production and Education

**DOI:** 10.1155/2022/4806763

**Published:** 2022-02-18

**Authors:** Honghai Li, Hongtao Deng, Yi Zhang

**Affiliations:** ^1^Northwest Normal University, Lanzhou, China; ^2^Physical Education Department, Xi'an University of Finance and Economics, Xi'an, Shaanxi, China; ^3^School of Management, Xi'an University of Finance and Economics, Xi'an, Shaanxi, China

## Abstract

This study aims to arouse students' interest in physical education (PE) in response to President Xi Jinping's call to strengthen students' physical quality because cultural courses occupy PE classes. Problem-based learning (PBL) is introduced, and a new teaching method of PE is proposed based on the convolutional neural network (CNN) in deep learning (DL). This method is employed to teach the experimental subjects in solid ball throwing. The students' interest, learning ability, and physical quality in the solid ball are investigated by a questionnaire survey. The questionnaire survey shows that the students' academic performance in solid ball throwing is improved, and their problem-solving ability, group cooperation ability, and theory learning ability are improved. Their time on a 1000-meter long run is shortened, and their body flexibility is improved. Therefore, it is believed that this new teaching method based on DL plays a significant role in improving students' physical quality.

## 1. Introduction

Due to the increasing proportion of cultural classes in daily teaching activities, physical education (PE) classes are becoming fewer and fewer, resulting in the gradual decline of primary and secondary school students [1]. In the 2018 National Education Conference, President Xi Jinping announced that it is necessary to pay attention to students' physical quality [2]. Because of insufficient physical exercise, the arm strength of primary and secondary school students is weak, and many students' arm strength tests cannot meet the qualified indexes. Therefore, it is time to enhance their arm strengths [3]. Throwing solid balls can significantly increase students' arm strength and improve their body flexibility [4]. With the development of science and technology, the traditional teaching method of PE is unable to meet the needs of students. Therefore, the traditional teaching method of PE is improved, and a new teaching method of solid ball training is proposed. The problem-based learning (PBL) method is used to explore various disciplines and has made some achievements. Here, it tries to be applied to solid ball teaching to improve the physical quality of primary and middle school students.

RETRACTED

PBL, as a teaching method in the new era, is discussed by many research experts in the teaching process of various subjects. Rahmawati et al. implemented a Hybrid-PBL model and applied it to the teacher's electronic modelling in the physics course. It has a good effect on arousing students' interest in study [5]. Susanti et al. used the PBL model to test junior high school students' mathematical communication ability and found it can improve their mathematical communication skills [6]. Boleng and Maasawet adopted the PBL teaching method to teach students cooperative scripts. They found that the PBL teaching method has a significant impact on improving students' critical thinking and can be applied to teaching literature [7]. Zhou found that the PBL teaching method can improve students' analytical, openness, and fairness qualities and their explanatory abilities in learning English [8]. These research results show that the PBL teaching method meets the needs of the times and can accurately improve the teaching quality of different subjects. However, many students are reluctant to take physical exercise because of laziness. Therefore, how to inspire students' interest in doing sports and improve the efficiency of classroom teaching are significant problems that need to be solved. Under this circumstance, the convolutional neural network (CNN) is combined in deep learning (DL), and a new teaching method based on PBL is proposed [9]. Aji et al. explored the effectiveness of PBL on basketball playing. According to the descriptive statistical results, more and more achievements have been made. PBL is effective for basketball playing through audio-visual media [10]. Pyle and Hung discussed the influence of PBL on students' motivation based on phonetics science courses. They revealed the influencing factors of emotional characteristics, such as emotion and personal-psychological connection. They found that these were often underestimated in the PBL design [11]. After the method is used, students can actively participate in the PE classes, realizing the unity of knowledge and action in the teaching process.

PBL is designed based on CNN in DL. Based on the technique, two classes of students in two middle schools in a particular place are investigated to solve the problem that physical education (PE) in primary and secondary schools is reduced and the students' physical quality is declining. CNN in DL is combined with PBL to explore how to arouse students' interest in learning solid ball throwing. Students' physical fitness indexes are tested before and after the solid ball training to discuss whether this new teaching method can be used in PE. The concept of PBL is summarized, and the relevant theory of CNN in DL is expounded. And a new teaching plan is proposed based on DL and PBL. After that, the physical fitness indexes of the students are investigated by a questionnaire survey to judge whether this teaching method is feasible. The specific process is as follows: (1) the research background is introduced, and the relevant literature is reviewed to explain the research purpose and plans. (2) The related concepts of PBL are described, and DL's learning steps and procedures are displayed. (3) CNN in DL is used to establish the PBL teaching strategy, and a questionnaire is designed for students' opinions on the PBL teaching method. (4) The questionnaire survey data are analyzed, and the test of students' physical indexes is carried out to explore the performance of PBL. The innovation is to combine the neural network in DL with PBL. On this basis, the student's interest in the course and their academic achievements are discussed, making the research results universal. PBL can inspire students' interest, improve their learning ability, help them easily acquire the throwing skill of solid balls, and strengthen students' physical quality.

RETRACTED

## 2. Materials and Methods

### 2.1. Theory and Characteristics of PBL

PBL is a problem-based learning method. Howard Barrows put forward and defined it as a kind of problem analysis method in the learning process [12]. It is student-centered, and teachers are responsible for guiding students and arousing their interest in learning in a scenario.

PBL is not didactic. In the teaching process, the questions raised by teachers are the learning content, and the answers are in the questions. Then, the students are divided into small groups to discuss the questions independently and find the answers. The teaching process by using PBL is shown in Figure 1. Teachers are required to give a topic and raise some questions about it. They are also responsible for leading in the topic's content and analyzing the questions for independent learning and discussion. After discussion, the group leader of each group is selected to explain their group's views to the class, and the teachers give some comments on their answers.

The PBL teaching method has four characteristics [13], as shown in Table 1. It takes students as the main body in the classroom rather than the classroom content led by teachers. Different from the traditional teaching method, PBL focuses on dividing students into groups for learning and discussion.

The PBL teaching method falls into four links, as shown in Table 2 [14], which are scenario setting, analysis, solution, and evaluation.

PBL being widely used in course teaching is a tremendous advantage that traditional teaching methods do not have. For example, the teaching content of PE is demonstrated by teachers and imitated by students using the conventional teaching method, and teachers correct students' imitated acts. If the teaching mode is used repeatedly, students gradually lose interest in the course. In addition, it ignores students' differences, personality development, and the interaction between teachers and students, resulting in a harmful learning effect [15].  Figure 2 shows the procedure of traditional teaching methods.

RETRACTED

Integrating the PBL teaching method and solid ball teaching also needs to be analyzed. Throwing the solid ball can exercise students' explosive force and improve coordination. The traditional teaching method makes it easy to make students lose interest in throwing the solid ball. Learning it is also severe, resulting in poor learning effects. The PBL teaching method updates the traditional teaching method and arouses students' interest in learning in a new environment [16].  Table 3 shows the difference between the PBL and traditional teaching methods.

Moreover, as one of the sports in the high school entrance examination in China, throwing the solid ball also needs to be paid more attention to. And necessary training should be given to solid ball throwing if you want to score high.

In the current reform of primary and middle school students' education, PE is the top priority, and it attaches importance to students' morality and physical quality. The PBL teaching method cultivates students' specialty and improves students' cooperation and communication ability. The PBL teaching method is widely used in school curriculum education, medicine, health, and other related fields. For example, the PBL teaching method effectively helps students pick up medical knowledge in treatment. It is also used in tourism vocational education to improve the learning effect. In addition, it can even be applied to fashion design [17–19].

### 2.2. Theory of DL

DL is a learning method that pays attention to learners' motivation, knowledge, concept, state, result, and thinking. According to the learning tasks, teachers should guide students to perform DL meaningfully and express their ideas [20]. Shallow learning is to make learners get a simple, low-level cognitive process. At the same time, DL is the integration of fragmented information by combining various disciplines of knowledge to establish a bridge between new and old knowledge, promoting the students' understanding and application of knowledge. DL has several features, as shown in Table 4 [21].

Due to the influence of motivation, DL has a clear route and an open perspective. It is divided into three stages: the first stage is the introduction, which takes learning as the primary way to obtain theoretical knowledge [22]; the second is the main body, in which knowledge is integrated, and the mistakes are analyzed, thereby improving their judgment ability and doubting ability [23]; the third is the evaluation stage; a positive and good learning atmosphere is created through mutual evaluation or self-evaluation between teachers and students in the same group, having a correct attitude towards study [24]. The process of DL is shown in Figure 3. After the subjects are given the topic, they activate the relevant knowledge in their minds, discuss the topic using the previous knowledge, build a bridge between existing and new knowledge, and make the topic logical, creating a new knowledge system.

RETRACTED

### 2.3. CNN in DL

CNN includes the input layer, the hidden layer, and the output layer. The input layer is responsible for conveying the data to the neural network for operation, and the output layer exports the completed data to the following link. The hidden layer, including many levels, is used for data processing [25]. The structure of CNN is shown in Figure 4.

(1) Local response normalization [26] is the most common algorithm in CNNs. The response value is calculated by

(1) $$\begin{array}{c} b_{x,y}^{i}=\frac{a_{x,y}^{i}}{{\left(k+\alpha \sum_{j=\text{max}\left(0,i-\left(n/2\right)\right)}^{\text{min}\left(N-1,i+\left(n/2\right)\right)}{\left(a_{x,y}^{i}\right)}^{2}\right)}^{\beta }}. \end{array}$$

*a*_*x*,*y*_^*i*^ is the value of the first input at coordinates (*x*, *y*), *N* is the number of input data, and *n* is the normalization of adjacent *n* data. *n*, *α*, and *β* are adjustable parameters, and their general values are 5, 0.0005, and 0.5.

*a*_*x*,*y*_^*i*^ is the value of the *i*-th input at coordinate (*x*, *y*), *N* is the number of input data, and *n* is the mean square error (MSE) of normalizing the adjacent *n* data. *n*, *α*, and *β* are adjustable parameters, and their values are 5, 0.0005, and 0.5.

In deep CNNs, decision operations are needed, and the standard strategy is used as the decision layer. If there are *N* kinds of data and the classifier contains N output points corresponding to the discrete probability distribution *p*_*i*_, ∑*p*_*i*_=1. *h* represents the input feature vector of the classifier, and *W* is the weight, then if there are *N* kinds of data, the classifier contains *N* output points corresponding to a discrete probability distribution *p*_*i*_, so that ∑*p*_*i*_=1. If *h* is the input feature vector of the classifier and *W* is the weight, then

(2) $$\begin{array}{c} p_{i}=\frac{\text{exp}\left(\sum_{k}h_{k}W_{k},i\right)}{\sum_{j=1}^{N}\text{exp}\left(h_{k}W_{k},i\right)}. \end{array}$$

In (2), *p*_*i*_ is the discrete probability distribution, *W* is the weight value, and *h* is the gradient. The type of prediction is expressed as

(3) $$\begin{array}{c} c={\text{arg}}_{j}\text{max}p_{i}. \end{array}$$

The cost function of the classifier is

(4) $$\begin{array}{c} J\left(W\right)=-\frac{1}{m}\left[\overset{m}{\underset{i=1}{\sum }}\overset{N}{\underset{j=1}{\sum }}1*\left\{y^{i}=j\right\}\text{log}\frac{e^{W_{j}^{T}h^{\left(i\right)}}}{\sum_{l=1}^{N}e^{W_{j}^{T}h^{\left(i\right)}}}\right]. \end{array}$$

*W*_*j*_^*T*^ *h* ^(*i*)^ is the gradient of *J*(*W*), and the gradient of parameter *W* can be obtained by CNN.

RETRACTED

*W*_*j*_^*T*^ *h* ^(*i*)^  is the gradient of *J* (*W*), and then the gradient of parameter *W* can be obtained by using CNN.

In DL, the support vector algorithm converts low-dimensional classification into high-dimensional space by introducing a kernel function. Linear regression and nonlinear regression belong to the support vector machine (SVM) regression. In linear regression, the function is calculated by

(5) $$\begin{array}{c} f\left(x\right)=\omega \cdot x+b. \end{array}$$

It is necessary to find *ω* to ensure the calculation ability of the equation. If there exists function *f*, it can estimate (*x*_*i*_, *y*_*i*_) in precision *ε*. Solving *ω* becomes a convex optimization problem, and the equations are

(6) $$\begin{array}{c} {\text{min}}_{\omega ,b,\xi ,\xi^{*}}\frac{1}{2}\omega^{T}\omega +c\overset{n}{\underset{i=1}{\sum }}\left(\xi +\xi^{*}\right),\\ \xi^{*}=\left\{\begin{array}{c} 0,f\left(x_{i}\right)-y_{i}\leq \varepsilon ,\\ \left|f\left(x_{i}\right)-y_{i}\right|-\varepsilon ,\left|f\left(x_{i}\right)-y_{i}\right|\geq \varepsilon . \end{array}\right. \end{array}$$

In equation (6), *c* is a penalty factor. In solving optimization problems, *c* is a fixed penalty factor, and it represents the penalty strength of the model for data beyond interval *ε*. Equation (6) is used to transform the problem into the quadratic programming problem by using the duality principle, and a Lagrange equation is established, as shown in equation (8):

(7) $$\begin{array}{c} l\left(\omega ,\xi_{i},\xi_{i}^{*}\right)=\frac{1}{2}\|\omega {\|}^{2}+C\left(\overset{m}{\underset{i=1}{\sum }}\xi_{i}+\xi_{i}^{*}\right)-\overset{\infty }{\underset{i}{\sum }}\alpha_{i}\left(\varepsilon +\xi_{i}-y_{i}+\left(\omega \cdot x_{i}\right)+b\right)\\ -\overset{\infty }{\underset{i}{\sum }}\alpha_{i}^{*}\left(\varepsilon +\xi_{i}-y_{i}-\left(\omega \cdot x_{i}\right)-b\right)-\overset{m}{\underset{i=1}{\sum }}\eta_{i}\xi_{i}+\eta_{i}^{*}\xi_{i}^{*}. \end{array}$$

In (7), if the partial derivatives of *ω*, *b*, *ξ*_*i*_,  and *ξ*_*i*_^*∗*^ are 0, the equations are transformed as

(8) $$\begin{array}{c} \frac{\partial l}{\partial \omega }=\omega -\overset{m}{\underset{i=1}{\sum }}\left(\alpha_{i}-\alpha_{i}^{*}\right)x_{i}=0,\\ \frac{\partial l}{\partial b}=\overset{m}{\underset{i=1}{\sum }}\left(\alpha_{i}-\alpha_{i}^{*}\right)=0,\\ \frac{\partial l}{\partial \xi_{i}}=C-\alpha_{i}-\eta_{i}=0,\\ \frac{\partial l}{\partial \xi_{i}^{*}}=C-\alpha_{i}^{*}-\eta_{i}^{*}=0. \end{array}$$

The dual optimization problem is solved by simplifying equations (8), as shown in the following equations:

(9) $$\begin{array}{c} \min\frac{1}{2}\overset{m}{\underset{i,j=1}{\sum }}\left(\alpha_{i}-\alpha_{i}^{*}\right)\left(\alpha_{j}-\alpha_{j}^{*}\right)x_{i},x_{j}+\overset{m}{\underset{i=1}{\sum }}\alpha_{i}\left(\varepsilon -y_{i}\right)+\overset{m}{\underset{i=1}{\sum }}\alpha_{i}^{*}\left(\varepsilon +y_{i}\right), \end{array}$$

(10) $$\begin{array}{c} s.t.\;\left\{\begin{array}{c} \overset{m}{\underset{i=1}{\sum }}\left(\alpha_{i}-\alpha_{i}^{*}\right),\\ \alpha_{i},\alpha_{i}^{*}\in \left[0,C\right]. \end{array}\right. \end{array}$$

*ω* can be obtained by equations (9) and (10):

(11) $$\begin{array}{c} \omega =\overset{N}{\underset{i=1}{\sum }}\left(a_{i}+a_{i}^{*}\right)x_{i}. \end{array}$$

According to the Lagrange theorem, the relationship of equations (12), (13), and (14) is

(12) $$\begin{array}{c} a_{i}\left(\varepsilon +\xi_{i}-y_{i}+\omega x+b\right)=0, \end{array}$$

(13) $$\begin{array}{c} a_{i}^{*}\left(\varepsilon +\xi_{i}^{*}-y_{i}+\omega x+b\right)=0, \end{array}$$

(14) $$\begin{array}{c} \left\{\begin{array}{c} \xi_{i}\left(C-a_{i}\right)=0,\\ \xi_{i}\left(C-a_{i}^{*}\right)=0. \end{array}\right. \end{array}$$

In addition, the relationship shown in equation (15) can be obtained:

(15) $$\begin{array}{c} \omega =\overset{m}{\underset{i=1}{\sum }}\left(\alpha_{i}-\alpha_{i}^{*}\right)x_{i}, \end{array}$$

*f*(*x*) presents the relationship shown in the following equation:

(16) $$\begin{array}{c} f\left(x\right)=\sum \left(\alpha_{i}-\alpha_{i}^{*}\right)x_{i}\cdot x+b. \end{array}$$

Generally speaking, linear regression is calculated under ideal conditions. But in actual prediction, there are many influencing factors, and the kernel function maps the sample into high-dimensional space. The optimization can be achieved by the following equations:

(17) $$\begin{array}{c} \omega \left(a,a^{*}\right)=-\frac{1}{2}\overset{N}{\underset{i,j=1}{\sum }}\left(a_{i}-a_{i}^{*}\right)\left(a_{j}-a_{j}^{*}\right)K\left(x_{i},x_{j}\right)+\overset{N}{\underset{i=1}{\sum }}\left(a_{i}-a_{i}^{*}\right)y_{i}-\overset{N}{\underset{i=1}{\sum }}\left(a_{i}+a_{i}^{*}\right)\varepsilon , \end{array}$$

(18) $$\begin{array}{c} \overset{N}{\underset{i=1}{\sum }}\left(a_{i}^{*}-a_{i}\right)=0, \end{array}$$

(19) $$\begin{array}{c} 0\leq a_{i},a_{i}^{*}\leq \frac{C}{N},i=1,2,\ldots ,N. \end{array}$$

The relationship of equations (17), (18), and (19) is solved, and equations (20) and (21) are obtained:

(20) $$\begin{array}{c} \omega =\overset{N}{\underset{i=1}{\sum }}\left(a_{i}^{*}-a_{i}\right)\phi \left(x_{i}\right), \end{array}$$

(21) $$\begin{array}{c} b=y_{i}-\overset{N}{\underset{i=1}{\sum }}\left(a_{i}^{*}-a_{i}\right)K\left(x_{i},x_{j}\right)-\varepsilon . \end{array}$$

Regression functions are calculated by the following equations:

(22) $$\begin{array}{c} f\left(x\right)=\overset{N}{\underset{i=1}{\sum }}\left(a_{i}-a_{i}^{*}\right)\left(\phi \left(x_{i}\right)\cdot \phi \left(x\right)\right)+b, \end{array}$$

(23) $$\begin{array}{c} f\left(x\right)=\overset{N}{\underset{i=1}{\sum }}\left(a_{i}-a_{i}^{*}\right)k\left(x_{i}\cdot x\right)+b. \end{array}$$

In addition, the calculation can be achieved according to BPNN. BPNN completes the infinite closed mapping from *n*-dimensional to *m*-dimensional space vector. If the transfer function of the hidden layer is *f*_1_(.) and that of the output layer is *f*2(.), then

(24) $$\begin{array}{c} z_{k}=f_{1}\left(\overset{n}{\underset{i=0}{\sum }}v_{ki}x_{i}\right),\;k=1,2,\ldots ,q,\\ y_{j}=f_{2}\left(\overset{n}{\underset{k=0}{\sum }}w_{jk}z_{k}\right),\;j=1,2,\ldots ,m. \end{array}$$

In the back propagation, the number of *x*_1_, *x*_2_,…, *x*_*p*_ is set to *P*, and *y*_*j*_^*p*^(*j*=1,2,…, *m*) can be obtained after the input network. The error function is square, and the error result of the *p* sample is *Ep*:

(25) $$\begin{array}{c} E_{P}=\frac{1}{2}\overset{m}{\underset{j=1}{\sum }}{\left(t_{j}^{p}-y_{j}^{p}\right)}^{2}. \end{array}$$

In equation (25), *t*_*j*_^*p*^ is the expected output. For the total number of samples P, the global error is calculated by

(26) $$\begin{array}{c} E=\frac{1}{2}\overset{P}{\underset{p=1}{\sum }}\overset{m}{\underset{j=1}{\sum }}\left(t_{j}^{p}-y_{j}^{p}\right)=\overset{P}{\underset{p=1}{\sum }}E_{P}. \end{array}$$

The weight value of the output layer changes and *w*_*jk*_ is adjusted by the cumulative error by BP to reduce global error *E*, as shown in the following equation:

(27) $$\begin{array}{c} \Delta w_{jk}=-\eta \frac{\partial E}{\partial w_{jk}}=-\eta \frac{\partial }{\partial w_{jk}}\left(\overset{P}{\underset{p=1}{\sum }}E_{P}\right)=\overset{P}{\underset{p=1}{\sum }}\left(-\eta \frac{\partial E_{P}}{\partial w_{jk}}\right). \end{array}$$

In equation (27), *η* is the learning rate. The following equation defines the error signal:

(28) $$\begin{array}{c} \delta_{yj}=\frac{\partial E_{p}}{\partial S_{j}}=\frac{\partial E_{p}}{\partial y_{j}}\cdot \frac{\partial y_{j}}{\partial S_{j}}. \end{array}$$

Based on the chain theorem, equation (28) can be written as follows:

(29) $$\begin{array}{c} \frac{\partial E_{p}}{\partial S_{j}}=\frac{\partial E_{p}}{\partial y_{j}}\cdot \frac{\partial y_{j}}{\partial S_{j}}=-\delta_{yj}z_{k}=-\overset{m}{\underset{j=1}{\sum }}\left(t_{j}^{p}-y_{j}^{p}\right)f_{2}^{\prime }\left(S_{j}\right)z_{k}. \end{array}$$

Therefore, the final weight of each neuron in the output layer can be adjusted by the following equation:

(30) $$\begin{array}{c} \Delta w_{jk}=\overset{P}{\underset{p=1}{\sum }}\overset{m}{\underset{j=1}{\sum }}\left(t_{j}^{p}-y_{j}^{p}\right)f_{2}^{\prime }\left(S_{j}\right)z_{k}. \end{array}$$

The hidden layer's weight changes and is similar to that of the output layer. Equation (31) can be obtained:

(31) $$\begin{array}{c} \Delta v_{ki}=\overset{P}{\underset{p=1}{\sum }}\overset{m}{\underset{j=1}{\sum }}\eta \left(t_{j}^{p}-y_{j}^{p}\right)f_{2}^{\prime }\left(S_{j}\right)w_{jk}f_{1}^{\prime }\left(S_{k}\right)x_{i}. \end{array}$$

RETRACTED

### 2.4. Experiment Design of the PBL Teaching Method Based on DL

Figure 5 shows the flow of the experiment. The experiment is carried out in two middle classes in a particular school. The two classes are randomly selected. One class is the experimental group in which the PBL method is used to teach the students, and the other class serves as the control group in which the students are guided by the traditional teaching method. After the experiment, the physical indexes of the students are tested and compared, and their performance is evaluated.

### 2.5. Questionnaire on the Solid Ball Training for Primary and Secondary School Students

Through literature review and comparative analysis, a set of tests are conducted for primary and middle school students before and after the solid ball training, and the effect of the proposed teaching method is analyzed. The details of the questionnaire are shown in Table 5 [27].

In the experimental environment, the students who take the solid ball course in a school are investigated, and the teaching content of the two groups is the same.

After the questionnaire design is completed, it is necessary to evaluate its validity. The validity of the questionnaire is tested [28], and the evaluation analysis is shown in Table 6.

After the evaluation, it is found that the questionnaire has high validity and can be used for this experiment. Two months later, 200 questionnaires are distributed to two middle schools, and 178 questionnaires are collected after the incomplete and damaged questionnaires are excluded. 160 valid questionnaires are collected, including 75 valid questionnaires in middle school A and 85 in middle school B. The results of the two middle schools are compared, and the comparative results are analyzed by using SPSS statistical software for a *t*-test [29]. The scores of the answers to the questions are calculated.

RETRACTED

Hypothesis (1): the new teaching method based on DL can effectively arouse students' interest in solid ball training and improve their communication and problem-solving abilities.

Hypothesis (2): the PBL teaching method based on DL can effectively improve students' teaching quality and physical quality.

### 2.6. Statistical Software

Statistical Package for the Social Sciences (SPSS) is used for statistical analysis and operation, data mining, predictive analysis, and decision support tasks. It is the earliest statistical software globally that uses a graphical menu-driven interface. Its most prominent feature is that the operation interface is highly supportive and has satisfactory output results. It displays almost all functions in a unified and standardized interface, uses windows to demonstrate the roles of various data management and analysis methods, and displays multiple function options in the dialog box.

It can provide many nonlinear modelling tools and multidimensional scale analyses to help researchers carry out regression analysis. It liberates the data from data constraints, conveniently divides the data into two groups, establishes controllable models and expressions, estimates nonlinear models' parameters, and shows better prediction models than simple linear regression models. The following coefficients and parameters are included.

The samples are selected from a collection of measured values of some observation units. Sampling is based on the principle of randomization. Every observation unit in the population has the same opportunity to be selected, avoiding the impact of error and bias on the research results. The observation unit included in the sample is called the sample content or sample size, also known as the number of samples. Researchers measure and observe the feature of each observation unit, which is called a variable. The measured values of variables are called variable values or observed values, also known as data. The differences between individuals are called variations. Frequency is the number of data in each segment. The frequency distribution types include left skew and right skew. Median refers to the value in the middle after a group of values are ranked from small to large. Range, full range *R*, describes the distribution range of data. An extensive range indicates that the data distribution is scattered, and standard deviation S can reflect the dispersion of data distribution.

RETRACTED

## 3. Results

### 3.1. Comparison of Students' Interest in Solid Ball Courses

After the questionnaires are collected, SPSS is used to calculate the scores. Due to a large amount of data, the average score is used to evaluate the results. A total of four results are counted, including students' ability to analyze and solve problems, their ability to cooperate within the group, their ability to learn theories, and their interest in solid ball training. The statistical results are shown in Figure 6.

Figure 6 shows that students' problem-solving ability, group cooperation ability, learning ability, and learning interest are improved after two months' teaching by using the PBL teaching method based on DL. It is found that the scores of the students' problem-solving ability in the experiment group are about 5.73 points higher than those in the control group. Their scores of group cooperation ability are improved by 5.09 points higher than those in the control group. Their scores of theoretical knowledge are about 8.07 points higher than those in the control group, and the scores of learning interest are about 9.87 points higher than the control group. Compared with the students without using the PBL teaching method, the results show that the new teaching method based on DL can effectively arouse students' interest in the study and improve their learning ability. It can replace the traditional teaching methods.

### 3.2. Test on Students' Physical Quality

The teaching results and the reliability of the PBL teaching method are evaluated by testing students' physical fitness indexes and physical quality. The results are shown in Figure 7, and the test items are their heights, arm lengths, weights, 1000-meter races, and body forward bending.

In terms of height, the experimental group is on average 1 cm higher than the control group. The experimental group is about 2 cm higher than the control group in arm length. The experimental group is about 1.69 kg lighter than the control group in weight. The speed of the 1000 m long run of the experimental group is about 0.6 min faster than the control group. The experimental group is approximately 0.43 cm higher than the control group regarding body forward bending. The data show that the physical quality of the students who received the solid ball training by PBL based on DL is higher than the students by using the traditional teaching method. And their heights and arm length increase, while those of the students in the other class decrease, indicating that the student's physical quality in class A is enhanced. The time the students spent on the 1000-meter race is shortened, showing that the students' cardiopulmonary ability is improved. The increase in the length of the body forward bending demonstrates that the flexibility of the students' bodies is improved. This shows that the new teaching method based on DL can concentrate students' attention after students' interest is aroused. The method proposed can help students obtain more comprehensive exercises and improve their physical quality compared with traditional teaching methods. This also shows the advantages of the new PBL teaching method.

RETRACTED

## 4. Discussion

After the experiment, the results are summarized, compared, and analyzed. Through the PBL teaching strategy, students' interest in the solid ball course is inspired, their learning enthusiasm surges upward, and their physical quality is also enhanced. From the tests of height, weight, arm length, and body forward bending, the scores of the students in the experimental group are higher than before. Simonton et al. adopted the PBL teaching method to discuss how PBL affects students' learning experience, and uttered that more research should be encouraged on the design and implementation of PBL in PE [30]. Ran et al. [31] found that the K-means clustering algorithm can cluster the data and capture the data hotspots. The research results are similar to the expected. It is believed that PBL can be applied to students' PE and provide some opinions for intelligent education.

## 5. Conclusions

In the current teaching schedule of primary and secondary courses, PE classes are gradually reduced due to the increasing proportion of cultural courses, and the traditional teaching methods cannot effectively evoke students' interest in learning. Therefore, a teaching method based on PBL and DL is proposed. After two months' teaching, a questionnaire is used to explore the teaching effect of the new teaching method. Through the analysis of the data of the questionnaire, it is found that the teaching method based on PBL and DL can effectively inspire students' interest in solid ball throwing. The physical qualities of the students who are taught by the method based on PBL and DL are higher than those who are taught by the traditional teaching method. The height and arm length increase and the weight decreases, indicating that the physical development of the students is enhanced. Their time spent on 1000-meter running is shortened, indicating that the students' cardiopulmonary ability is improved. The increase in the length of forwarding flexion in the sitting position shows that the flexibility of students' bodies is improved. Therefore, this PBL physical education teaching method plays a significant role in students' solid ball courses. It arouses students' interest in learning the course and helps students master the key points of throwing skills, so that students' relevant physical indexes are significantly improved. The research provides a basis for establishing the intelligent education system and a reference for improving the teaching method for other courses. After the experiment, the students' feelings can also be investigated. This proves that the experimental results are comprehensive, the accuracy of the model experiment is high, and the time-sensitivity of the model is also high. However, there are still some shortcomings that need to be improved. For example, the size of experimental samples is too small and individual differences are not excluded; the physical quality of some students is better than that of most students before the experiment. In the follow-up research work, the variables should be controlled before the experiment, and the students with a small score gap in PE tests should be regrouped. This can further prove the universality of the PBL teaching model. Therefore, in the subsequent research, the size of test subjects will be expanded and the experiment results will be more universal.

RETRACTED

PE is cut down in the courses of primary and secondary schools because educators pay more attention to the cultural courses and neglect the importance of PE, which weakens the students' physical quality. In addition, the traditional teaching methods of PE cannot effectively stimulate students' interest, and the actual teaching quality is not satisfactory. Under this condition, a PBL teaching method is proposed based on CNN in DL. And it is used to teach the students in two middle schools to play a solid ball. After the training, a questionnaire survey is conducted to investigate their performance and physical qualities. The results show that the PBL teaching method can arouse students' interest in solid ball courses, and their physical qualities are significantly improved. Therefore, it is concluded that the PBL teaching method can be applied to PE and even other courses. However, there are still some shortcomings that need to be improved. For example, the sample size is small, which may affect the research conclusions. Furthermore, the physical qualities of some students are better than others before the experiment, and there are also some exceptional cases in the investigation. In view of these, the number of research subjects will be expanded and more in-depth analysis will be made in the subsequent study.

RETRACTED

## Figures and Tables

**Figure 1:** Teaching process by using PBL.

**Figure 2:** Procedure of traditional teaching methods.

**Figure 3:** Process of DL.

**Figure 4:** Structure of CNN.

**Figure 5:** Process of the experiment.

**Figure 6:** Scores of students' results.

**Figure 7:** Test results of students' physical fitness.

**Table 1:** Characteristics of the PBL teaching method.

Characteristics	Content
The questions are orientated.	Students can discuss the questions with their imagination and knowledge. There are no fixed answers, so students must improve their ability to analyze the questions. Teachers or students can design the questions.
It is student-centered.	Teachers just need to raise questions or guide the direction of the discussion, and students should think about the answers to the questions and solve the problems encountered in the teaching process.
Students learn knowledge independently.	Students can think about how to learn, what to know, and where to learn. All the students should explore the most effective way in their learning process.
Students learn knowledge in groups.	Students can team up actively in the face of too complex problems and simplify complex issues through mutual assistance and task division. Within the group, they can exchange ideas and share achievements.

**Table 2:** PBL links.

Teaching links	Content
Scenario	Teachers design scenarios, ask questions, and display them through texts, pictures, audios, or videos
Analysis	Students analyze the questions, organize the thinking process, and decide whether to discuss in groups or by themselves
Solution	According to the design or group division, team members collect, collocate, analyze, and process the data in communication, idea exchange, and solution proposal
Evaluation	Individuals or group members show the results, explain their ideas, and finally optimize their solving methods. And teachers summarize at last.

**Table 3:** Differences between the PBL teaching method and traditional teaching methods.

The teaching methods	Learning form	Center	Teaching measures	Interaction degree	Teaching forms	Attitudes towards mistakes in the learning process	Teacher's roles	Students' knowledge	Knowledge chain
The PBL teaching method	Group learning	Student-centered	Improving students' skills	Interaction between students	Cooperation between students and teachers	Learning from the mistakes	The teacher only assigns the tasks	Students can master the skills they have learned	Students can use the knowledge and resources positively
Traditional teaching methods	All students are learning in a large class	Teacher-centered	Acquiring knowledge	Less interaction in the learning process	Teacher's lecture and instructions	Passively learning	Teachers deliver knowledge all the time	The knowledge learned is quickly forgotten	Learning tasks are the only teaching resources

RETRACTED

**Table 4:** Characteristics of DL.

Characteristics	Content
Student-centered	Learners are responsible for themselves and interested in the study. They can improve their learning quality and effect, and teachers guide the students to meet their needs.
Lifelong learning	Shallow learning only focuses on the immediate task and lacks reflection and evaluation for learning effects. DL requires timely correctness in understanding and constantly improves students' proficiency in knowledge.
Understanding ability	Shallow learning is passive learning, while DL focuses on understanding and solving problems with a skeptical attitude, which can help evaluate their learning effects and improve their profound thinking ability.
Integration ability	DL emphasizes integrating new and old knowledge and helps acquire knowledge more widely and establish their knowledge bases
Transformation ability	It can improve their self-understanding abilities, self-examination, self-evaluation, self-control, and transformation and summarize the knowledge learned
Application ability	Shallow learning only solves immediate problems mechanically, while DL teaches students to solve problems using their knowledge
Problem-solving ability	Shallow learning can only solve problems with scattered knowledge, while DL emphasizes applying knowledge learned in real life to solve complex problems
Higher-order thinking	Shallow learning only focuses on low-level activities, such as understanding, memory, and recitation, while DL emphasizes high-level activities, such as application, analysis, evaluation, and creation

**Table 5:** Questionnaire on the solid ball training for primary and secondary school students.

Course	Classes	Grades
Survey on solid ball training	Questions	Rating
	In the classroom, I usually ask questions.	1 2 3 4 5
	In course training, I can find my own mistakes and correct them.	1 2 3 4 5
	I can correct my mistakes under teachers' guidance.	1 2 3 4 5
	I can find others' mistakes in cooperation.	1 2 3 4 5
	I can find my mistakes by comparison.	1 2 3 4 5
	I can think about action at different stages.	1 2 3 4 5
	I can consult the information of the solid ball and do some research in learning to throw the solid ball.	1 2 3 4 5
	I can actively find the difficulties.	1 2 3 4 5
	I am thinking actively in the theory course.	1 2 3 4 5
	I usually turn to teachers and students for help when I have trouble learning.	1 2 3 4 5
	I am willing to share my thoughts and ideas with my classmates.	1 2 3 4 5
	I actively communicate with group members.	1 2 3 4 5
	I actively help team members when they are in trouble.	1 2 3 4 5
	I usually actively display the results.	1 2 3 4 5
	I usually discuss with teachers about the difficulties.	1 2 3 4 5
	I usually express my opinions when classmates show theirs.	1 2 3 4 5
	I think solid ball training can help us have teamwork awareness.	1 2 3 4 5
	This teaching method can improve my communication skills.	1 2 3 4 5
Other		

RETRACTED

**Table 6:** Validity of the questionnaire.

Evaluation items	Rating		
	Highest (%)	Higher (%)	Lower (%)
Contents	30	62	8
Quantity	38	61	1
Structure	16	69	15

## Data Availability

The simulation and experimental data used to support the findings of this study are available from the corresponding author upon request.
